The article "A Deep Learning Model for Three-Dimensional Nystagmus Detection and Its Preliminary Application" was retracted in 2023. Reasons: compromised peer review; unreliable results or conclusions.

# A Deep Learning Model for Three-Dimensional Nystagmus Detection and Its Preliminary Application

**DOI:** 10.3389/fnins.2022.930028

**Published:** 2022-06-13

**Authors:** Wen Lu, Zhuangzhuang Li, Yini Li, Jie Li, Zhengnong Chen, Yanmei Feng, Hui Wang, Qiong Luo, Yiqing Wang, Jun Pan, Lingyun Gu, Dongzhen Yu, Yudong Zhang, Haibo Shi, Shankai Yin

**Affiliations:** ^1^Department of Otolaryngology—Head and Neck Surgery, Shanghai Jiao Tong University Affiliated Sixth People’s Hospital, Shanghai, China; ^2^IceKredit Inc., Shanghai, China; ^3^School of Computing and Mathematical Sciences, University of Leicester, Leicester, United Kingdom

**Keywords:** vertigo, nystagmus detection, benign paroxysmal positional vertigo, deep learning, neural network

## Abstract

Symptoms of vertigo are frequently reported and are usually accompanied by eye-movements called nystagmus. In this article, we designed a three-dimensional nystagmus recognition model and a benign paroxysmal positional vertigo automatic diagnosis system based on deep neural network architectures (Chinese Clinical Trials Registry ChiCTR-IOR-17010506). An object detection model was constructed to track the movement of the pupil centre. Convolutional neural network-based models were trained to detect nystagmus patterns in three dimensions. Our nystagmus detection models obtained high areas under the curve; 0.982 in horizontal tests, 0.893 in vertical tests, and 0.957 in torsional tests. Moreover, our automatic benign paroxysmal positional vertigo diagnosis system achieved a sensitivity of 0.8848, specificity of 0.8841, accuracy of 0.8845, and an F1 score of 0.8914. Compared with previous studies, our system provides a clinical reference, facilitates nystagmus detection and diagnosis, and it can be applied in real-world medical practices.

## Introduction

Of all the symptoms encountered clinically, vertigo is one of the most common complaints. Vertigo has a considerable impact on personal quality of life, which is exacerbated by aging (Neuhauser et al., 2005; Murdin and Schilder, 2015; Tonsen et al., 2016; Alyono, 2018). With a 12-month prevalence of 15–20% (Neuhauser, 2016), vertigo imposes a huge economic burden on primary health care with costs totalling 61.3 million pounds annually (Tyrrell et al., 2016; Kovacs et al., 2019). Unfortunately, the variety and heterogeneity of vestibular disorders greatly increases the difficulty in making a clinical diagnosis, leading to numerous repeat medical consultations with low rates of specific diagnoses (20–60%) and poor specialist referral rates (3–4%) (Kruschinski et al., 2008; Maarsingh et al., 2010a,b; Neuhauser, 2016). Unlike other diseases, vestibular disorders are difficult to diagnose due to the lack of typical signs and features.

The article "A Deep Learning Model for Three-Dimensional Nystagmus Detection and Its Preliminary Application" was retracted in 2023. Reasons: compromised peer review; unreliable results or conclusions.

Nystagmus, an involuntary, rapid, rhythmic, oscillatory eye movement, is the most important sign for the differential diagnosis of vestibular disorders (Eggers et al., 2019). There are three directions of nystagmus: horizontal, vertical, and torsional. Its detection is widely used in routine clinical evaluation of patients with vertigo in specialty clinics, via visual observation with the naked eye or video nystagmography (VNG) (Bhansali and Honrubia, 1999; Eggert, 2007). However, nystagmus recognition poses many challenges in modern clinical practice, including a lack of specialists and medical resources, complex and heterogeneous characteristics that are difficult to analyse, and sensitivity limitations in nystagmus recognition by the naked eye, especially when the nystagmus is subtle. In practice, it is difficult to evaluate patients with droopy eyelids or eyelashes covering their pupils using VNG, and the interference of infrared light and cosmetics around the eyes can make it worse (Ganança et al., 2010). Therefore, establishing a model for three-dimensional (3D) nystagmus detection is of great urgency.

With the advances in science and technology, a system for nystagmus detection could be achieved using artificial intelligence (AI). AI is an interdisciplinary subject dedicated to data-driven empirical learning (Wainberg et al., 2018) which has been considered a potential solution to several medical diagnostic challenges, especially in the fields of radiology and pathology. The accessibility, growth potential, and limited cost make AI a promising option for dealing with the lack of medical resources and specialists. The convolutional neural network (CNN) is one of the most widely used deep learning algorithms in AI-based applications, contributing to object classification, detection, and segmentation. This makes CNN promising for AI-based recognition of nystagmus due to its ability to capture specific features, extensive open-source codes, and the advanced research foundation for eye-tracking from other medical fields. However, pioneering research on CNN-based automated nystagmus detection encountered difficulty with pupil detection in some situations and fails to capture twisting eyeball movement. Still, there are proven object detection models (Szegedy et al., 2015, 2017) that have shown good performance in coping with the high frequency of noise (e.g., eye blink, head movements) faced in clinical practice. Currently, no nystagmus recognition system has been used for clinical diagnosis.

Benign paroxysmal positional vertigo (BPPV) is a common cause of vertigo and is diagnosed in 17–42% of patients with vertigo (Schappert, 1992; Katsarkas, 1999; Hanley et al., 2001). The BPPV diagnostic procedure costs approximately 2,000 USD, and 65% of patients undergo unnecessary diagnostic tests or therapeutic interventions (Wang et al., 2014). Since BPPV can be easily cured once correctly diagnosed, such a waste of resources could be avoided with an advanced diagnostic strategy. Notably, BPPV allows for different types of nystagmus to be observed in specific head positions and its characteristic nystagmus is relatively easy to analyse, offering a low threshold for AI diagnosis.

The article "A Deep Learning Model for Three-Dimensional Nystagmus Detection and Its Preliminary Application" was retracted in 2023. Reasons: compromised peer review; unreliable results or conclusions.

In this study, we developed an automatic system for detecting 3D eye movements based on deep learning. To improve the robustness and establish a reliable AI diagnostic system, we developed a new method to locate pupils accurately and detect iris twist. The model was validated in patients with BPPV and achieved high sensitivity and accuracy in nystagmus detection and disease diagnosis. In this study, we applied our model in BPPV diagnosis, not only as a real-world performance test of our algorithm model, but also in an attempt to develop an intelligent diagnostic system with real-world application potential.

## Materials and Methods

We enrolled patients from the outpatient clinic of the Department of Otolaryngology-Head and Neck Surgery of the Sixth People’s Hospital of Shanghai Jiao Tong University between September 2017 and November 2021 who underwent vestibular function tests using infrared video goggles (Verti Goggles-M, ZEHNIT Medical Technology, Shanghai, China). All patients complaining of symptoms of vertigo or dizziness would undergo two positional tests: the supine Roll Test and Dix-Hallpike manoeuvre. Each test lasted for at least 30 s until the end of eye movement. The recorded videos were labelled by three experts based on the BPPV diagnostic criteria of the Bárány Society (Von Brevern et al., 2015; Yao et al., 2018). The datasets for validation were selected with similar proportions of positive samples from the training data to avoid biased evaluation. The input data of our model were comprised of 1–4 clinical videos of each patient.

### Ethics Committee Approval

The study was approved by the Ethics Committee of Shanghai Sixth People’s Hospital and was conducted according to the Declaration of Helsinki. Written informed consent was obtained from all the participants. The study was registered in the Chinese Clinical Trials Registry (ChiCTR.org.cn) under the identifier ChiCTR-IOR-1711-506.

### Experimental Procedure

The overall framework of our diagnostic system is shown in Figure 1. Portable video goggles were adopted to capture pupil movement during the Dix-Hallpike manoeuvre and supine roll test. The procedure consisted of four parts: pupil detection, iris torsion measurement, the deep learning model, and disease inference.

The article "A Deep Learning Model for Three-Dimensional Nystagmus Detection and Its Preliminary Application" was retracted in 2023. Reasons: compromised peer review; unreliable results or conclusions.

**FIGURE 1:** Framework of the automatic nystagmus detection system. Procedures of our auto diagnosis system: pupil locator system, iris torsion measure, data pre-processing, CNN-based nystagmus detection model, and disease inference. CNN, convolutional neural network.

#### Pupil Locator

The raw clinic videos do not mark the position of the pupil centre; thus, the first step is to locate the pupil inside each frame. A pupil location algorithm was applied to locate the pupil centre in each video. Previous studies (Santini et al., 2018; Eivazi et al., 2019) have attempted to predict the parameters of pupil location using deep learning models. As the performance of deep learning algorithms continues to improve, pupil detection algorithms are often driven by data. Such data-driven models require a large amount of qualified data labelled by specialists, which is an expensive, slow, and error-prone manual process. To reduce the error and cost caused by annotation, we trained one deep-learning model with the architecture of Inception V4 (Szegedy et al., 2015, 2017) on an open-source dataset containing 66 high-quality, high-speed videos (Tonsen et al., 2016), and then used the pre-trained model to label our raw videos (Figure 2).

**FIGURE 2:** Objection detection model for pupil location. **(A)** Model architecture. **(B)** Feature extraction with different convolution kernels. **(C)** Visualisation of the pupil parameters: dot – pupil centre; circle – outer radius.

#### Torsional Movement Detection

Torsional nystagmus is a deterministic signal in BPPV diagnosis. Several methods have been proposed to measure the torsional movement (Wolberg and Zokai, 2000; Ojansivu and Heikkila, 2007; Alba et al., 2013) such as tracking stable iris features, template matching, and optical flow. We decided to use phase correlation techniques as our torsional measurement method, an approach that has typically been applied in image registration (Araujo and Dias, 1997; Abdullah-Al-Wadud et al., 2007).

The circular iris pattern was transformed by log-polar transformation. An image augmentation technique called histogram equalisation (Abdullah-Al-Wadud et al., 2007) was applied to extract slight features on iris pattern. Phase correlation, a frequency domain technique with broad applications in image alignment (Reddy and Chatterji, 1996), was used for the estimation of the similarity measure of two images (Figure 3).

**FIGURE 3:** Iris torsion measure. **(A)** Iris extraction. Circles: iris boundaries; rectangles: log-polar (left) and linear-polar transform (right). **(B)** Original and equalised histogram. **(C)** Iris patterns before and after equalisation. **(D)** Phase-only correlation function.

The article "A Deep Learning Model for Three-Dimensional Nystagmus Detection and Its Preliminary Application" was retracted in 2023. Reasons: compromised peer review; unreliable results or conclusions.

##### Log-Polar Transformation

The log-polar coordinate parameters ρ and θ denote the logarithmic radial distance from the pupil centre and the angle, respectively, corresponding to the radial distance from the centre and angle from the centre, respectively. Any point (x, y) in the original Cartesian plane can be reflected in the rectangular iris pattern (see computation below):


$$\begin{array}{c} \theta =a\,r\,c\,t\,a\,n\,\left(\frac{y-y\,0}{x-x\,0}\right)\,\#\,\left(1\right) \end{array}$$

$$\begin{array}{c} \rho =\text{log}\,\left(s\,q\,r\,t\,\left({\left(x-x\,0\right)}^{2}+{\left(y-y\,0\right)}^{2}\right)\right)\,\#\,\left(2\right) \end{array}$$

$$\begin{array}{c} X\,n\,e\,w=\frac{c\,o\,l\,s}{\text{log}\,\left(R_{m\,a\,x}\right)}\times \rho \,\#\,\left(3\right) \end{array}$$

$$\begin{array}{c} Y\,n\,e\,w=\frac{r\,o\,w\,s}{360}\times \theta \,\#\,\left(4\right) \end{array}$$

(X0, Y0) and (Xnew, Ynew) correspond to the centre of the pupil and coordinate mapping from the Cartesian domain to the rectangular iris pattern, respectively. Formulas (1) and (2) are used to calculate the log-polar coordinates of each point (x, y) in the Cartesian plane, and formulas (3)-(6) are used to resize the log-polar coordinates:


$$\begin{array}{c} \theta :\left[0^{o},360^{o}\right]->\left[0,c\,o\,l\,s-1\right]\,\#\,\left(5\right) \end{array}$$

$$\begin{array}{c} \rho :\left[0,R_{m\,a\,x}\right]->\left[0,r\,o\,w\,s-1\right]\,\#\,\left(6\right) \end{array}$$

Where *cols* and *rows* represent the scale of the image, and *Rmax* denotes the maximum radius sampled from the image.

##### Histogram Equalisation

We first calculated the probability mass function of all the pixels in the grayscale histogram of the original image using formula (7), where k represents the grayscale value and N_*k*_ represents the total number of pixels with grayscale k. Second, formula (8) generates the discrete cumulative distributive function. The transformed grayscale histogram is generated by formula (9). The contrast of the iris pattern was enhanced using histogram equalisation, which is useful for the further application of the phase correlation method.


$$\begin{array}{c} P\,M\,F\,\left(k\right)=\frac{N_{k}}{C\,o\,l\,s\times R\,o\,w\,s},k=0,1,2,255\,\#\,\left(7\right) \end{array}$$

$$\begin{array}{c} C\,D\,F\,\left(k\right)=\sum_{0}^{k}P\,M\,F\,\left(k\right)\,\#\,\left(8\right) \end{array}$$

$$\begin{array}{c} P\,i\,x\,e\,l_{n\,e\,w}\,\left(k\right)=255\times R\,o\,u\,n\,d\,\left(C\,D\,F\,\left(k\right)\right)\,\#\,\left(9\right) \end{array}$$

The article "A Deep Learning Model for Three-Dimensional Nystagmus Detection and Its Preliminary Application" was retracted in 2023. Reasons: compromised peer review; unreliable results or conclusions.

##### Phase Correlation

Several properties of Fourier transform, such as translation, rotation, reflection, and scale in the frequency domain, have been exploited for image registration. Phase correlation relies on the translation property of Fourier transform, based on estimating the shift between two images by calculating the maximum of the phase-only correlation function, which is defined as the inverse FFT of the normalized cross-spectrum between two images. Let f and g be the pixel signals of two images with displacement < dx, dy >, that is:


$$\begin{array}{c} g\,\left(x,y\right)=f\,\left(x-d\,x,y-d\,y\right)\,\#\,\left(10\right) \end{array}$$

Let the Fourier Transform function be:


$$\begin{array}{c} D\,F\,T\,\left(f\,\left(x,y\right)\right)=F\,\left(u,v\right)\,\#\,\left(11\right) \end{array}$$

D⁢F⁢T⁢(f⁢(x-d⁢x,y-d⁢y))=exp⁡(-i×2⁢π×(u⁢d⁢x+v⁢d⁢y)×F⁢(u,v))⁢#⁢(12)

The corresponding relationship of *F* and *G* is given by:


$$\begin{array}{c} G\,u,v=F\,\left(u,v\right)\times \exp\left(-i\times 2\,\pi \times \left(u\,d\,x+v\,d\,y\right)\right)\,\#\,\left(13\right) \end{array}$$

According to the properties of Fourier transform, the translational movement of the time-domain signal can be expressed by the phase difference in the frequency domain, which is equivalent to the phase of the cross-power spectrum:


$$\begin{array}{c} H\,\left(u,v\right)=\exp\left(-i\times 2\,\pi \times \left(u\,d\,x+v\,d\,y\right)\right)=\frac{F*\bar{G}}{\left|F*\bar{G}\right|}\,\#\,\left(14\right) \end{array}$$

The inverse Fourier transform of the phase difference is an impulse function, and the peak location calculated from formula (15) is the point of image registration.


$$\begin{array}{c} d\,x,d\,y=a\,r\,g\,m\,a\,x\,\left\{D\,F\,T^{-1}\,\left(H\,\left(u,v\right)\right)\right\}\,\#\,\left(15\right) \end{array}$$

The sharp peak appears only when two images have best matched the height which gives a similarity measure for image alignment. Also, the location of the peak represents the displacement between images, which is what we need to quantify the eye torsional movement between two consecutive frames.

In horizontal/vertical movements, the velocity curve was obtained by applying differencing to the time series of pupil centre coordinates, while the velocity in torsional dimensions was defined as the similarity measure between two consecutive frames (Figure 4). Due to the existence of noise frames in test videos caused by eye blinking, head shifting, and mistaken operations, we applied the DBSCAN method (an unsupervised machine learning algorithm that has excellent performance for detecting outliers) to eliminate the noise data.

The article "A Deep Learning Model for Three-Dimensional Nystagmus Detection and Its Preliminary Application" was retracted in 2023. Reasons: compromised peer review; unreliable results or conclusions.

**FIGURE 4:** Eye movement data generation. Each video was transformed to eye movement velocity in three dimensions. Horizontal and vertical velocity: coordinates of the pupil centre. Torsional velocity: the shift between two consecutive frames.

#### Deep Learning Model

We adopted several data augmentation technologies to enhance our model’s performance due to the insufficient amount of data for deep learning model training. We first split clinic videos into overlapping sub-samples with a fixed length (Figure 5A). Then, each video clip was horizontally and vertically reversed, and white noise data was added (Figure 5B). Finally, the over-sampling technique was applied to balance the labelled data in nystagmus and non-nystagmus. One-dimensional (1D CNN) was used as the architecture of our nystagmus detection model, an architecture that performed well in similar tasks (Yildirim et al., 2018; Zabihi et al., 2019). Patients labelled positive in the supine roll test showed horizontal nystagmus, while the Dix-Hallpike manoeuvre was applied to detect vertical/torsional nystagmus. We trained three models for horizontal, vertical, and torsional nystagmus detection (Figure 5C).

**FIGURE 5:** Data pre-processing and the deep learning model for nystagmus detection. **(A)** The rolling cut of the velocity curve to fix the length of the time series; sub-samples including a nystagmus pattern (marked as red) are labelled as positive (otherwise negative). **(B)** Data augmentation methods applied to generate new examples of nystagmus. Upper left: Original data with nystagmus signals. Upper right: Data flipped on the x-axis. Bottom left: Data flipped on the y-axis. Bottom right: Add white noise **(C)** shows the model structures. GMP, global max pooling; MLP, multi-layer perception.

#### Disease Inference

The variety and complexity of BPPV diseases increased the difficulty of automatic diagnosis. A decision tree procedure was thus established to determine the exact type of BPPV disease (Figure 6C), depending on the direction and duration of the nystagmus signal.

**FIGURE 6:** Disease diagnosis process. **(A)** Peak detection: all velocity peaks in two directions are detected. **(B)** The predicted labels of test data, longest consecutive positive sub-samples represent the position of nystagmus. **(C)** The decision tree that simulates the diagnosis of specialists.

##### Nystagmus Direction

The velocity peaks are detected from the time series (Figure 6A), then the median velocity is obtained in two directions. The direction with a larger absolute median value is determined to be the direction of nystagmus.

The article "A Deep Learning Model for Three-Dimensional Nystagmus Detection and Its Preliminary Application" was retracted in 2023. Reasons: compromised peer review; unreliable results or conclusions.

##### Nystagmus Duration

The prediction steps label each sub-sample in the test set, and the length of the longest consecutive positive segmentation is defined as the duration of nystagmus. Figure 6B shows an example. The test video is separated into 31 sub-samples for model prediction and the number of consecutive positive samples given by model prediction is 19; an estimate of nystagmus duration can be calculated with formula (16):


$$\begin{array}{c} N\,y\,s\,t\,a\,g\,m\,u\,s\,D\,u\,r\,a\,t\,i\,o\,n=\\ F\,r\,a\,m\,e\times N-O\,v\,e\,r\,l\,a\,p\times \left(N-1\right)-F\,r\,a\,m\,e\,\#\,\left(16\right) \end{array}$$

Where frame is the length of sub-samples (set as 400/600); N is the number of consecutive positive sub-samples; and overlap is the length of the overlapped part.

### Statistical Analyses

The sample size was determined by the total amount of high-quality labelled data collected. The lack of available data was the most significant challenge when applying deep learning algorithms for BPPV diagnosis; therefore, we used all the data to strengthen the performance, instead of performing a power analysis. The 854 patient cases were randomly selected from thousands of patients in the case pool and split into training, validation, and testing datasets by simple random sampling. The testing dataset was not available during modelling to ensure that the experimenters were blind to outcome assessment.

Statistical analysis was performed separately for the nystagmus detection model and BPPV disease inference to evaluate the overall performance of our automatic diagnosis system. For the primary datasets (training, validation, and test), binary classification evaluation was conducted by calculating the accuracy and area under the receiver operating characteristic curve (AUC) (which provides an aggregate measure of model performance at all classification thresholds) for each model in three directions. For disease inference, we computed the true positive (TP), false positive (FP), false negative (FN), true negative (TN), precision, recall accuracy, and F1 score at binary decision thresholds for the aggregate measure of the inference performance on different types of BPPV diseases.


$$A\,c\,c\,u\,r\,a\,c\,y=\frac{\left(T\,P+T\,N\right)}{T\,P+F\,P+F\,N+T\,N}$$

$$F\,1\,S\,c\,o\,r\,e=\frac{2\times P\,r\,e\,c\,i\,s\,i\,o\,n\times R\,e\,c\,a\,l\,l}{P\,r\,e\,c\,i\,s\,i\,o\,n+R\,e\,c\,a\,l\,l}$$

$$P\,r\,e\,c\,i\,s\,i\,o\,n=\frac{T\,P}{T\,P+F\,P}$$

$$R\,e\,c\,a\,l\,l=\frac{T\,P}{T\,P+F\,N}$$

## Results

### Participant Characteristics

We enrolled a total of 854 patients from the outpatient clinic of the Department of Otolaryngology-Head and Neck Surgery of the Sixth People’s Hospital of Shanghai Jiao Tong University between September 2017 and November 2021 who underwent vestibular function tests using infrared video goggles. We collected clinical videos from these patients’ records, including 3,496 horizontal movements and 5,962 vertical/torsional movements (Table 1). Among the 854 patients in our dataset, 304 (35.6%) were randomly selected as the training set, 93 (10.9%) were randomly selected as the validation set, 122 (14.3%) were selected as the testing set for nystagmus model performance evaluation, and the remaining 457 (53.5%, including the testing set previously mentioned) were selected to evaluate the accuracy of disease inference. To avoid data leaks, the split of training and validation datasets were determined by the patients, not clinical videos.

The article "A Deep Learning Model for Three-Dimensional Nystagmus Detection and Its Preliminary Application" was retracted in 2023. Reasons: compromised peer review; unreliable results or conclusions.

**TABLE 1:** Summary of the data sets (baseline).

	Sex (M/F)	Age (Mean ± SD)
**Training**		
LP	12/20	54.47 ± 5.28
RP	11/38	58.03 ± 13.44
LH	4/8	55.50 ± 17.28
RH	4/16	55.65 ± 15.21
LH cu	3/2	61.20 ± 12.79
RH cu	1/2	53.67 ± 27.43
Negative	54/129	47.52 ± 16.69
Total	89/215	51.16 ± 16.61
**Validation**		
LP	0/10	59.30 ± 15.71
RP	2/6	53.75 ± 16.18
LH	1/3	44.75 ± 12.61
RH	2/8	47.40 ± 14.32
LH cu	0/1	38.00
RH cu	0/2	78.50 ± 14.85
Negative	16/42	50.84 ± 15.42
Total	21/72	51.83 ± 15.74
**Testing**		
LP	19/24	52.00 ± 15.55
RP	31/69	53.60 ± 14.65
LH	4/21	54.12 ± 18.32
RH	19/36	57.23 ± 15.58
LH cu	6/10	52.06 ± 14.38
RH cu	7/3	46.20 ± 19.70
Negative	61/147	48.53 ± 18.09
Total	147/310	51.39 ± 16.98

*L, left; R, right; P, posterior semi-circular canal; H, horizontal semi-circular canal; cu, cupulolithiasis; M, male; F, female; SD, standard deviation.*

### Model Performance

Our model was trained to predict nystagmus in each single-frame segment. The model performance for identifying different types of nystagmus is summarised in Table 2. The AUC and accuracy of the horizontal and torsional models are shown in Figure 7. The overall performance of 502 cases from 457 patients (some cases taken by the same patient at a different visiting time) in terms of disease inference is shown in Tables 3, 4. The torsional model achieved a sensitivity and specificity of 0.8848 and 0.8841, respectively.

**TABLE 2:** Model performance in detecting horizontal, torsional, and vertical nystagmus.

	Horizontal	Torsional	Vertical
Cases	114	125	16
Samples	15,920	20,816	1,882
AUC	0.9825	0.9574	0.893
ACC	0.9303	0.8795	0.905

*AUC, area under curve; ACC, accuracy.*

**FIGURE 7:** Model performance. The receiver operating characteristic curve (ROC) of model performance classifying nystagmus types after model training. **(A)** The area under the ROC for measuring horizontal nystagmus is 0.982. **(B)** The area under the ROC for measuring torsional nystagmus is 0.957.

The article "A Deep Learning Model for Three-Dimensional Nystagmus Detection and Its Preliminary Application" was retracted in 2023. Reasons: compromised peer review; unreliable results or conclusions.

**TABLE 3:** One-vs-rest multi-class prediction results after symptoms inference.

		Model prediction						
		
		Negative	LP	RP	LH-ca	LH-cu	RH-ca	RH-cu
Doctor’s diagnosis	Negative	206	9	8	0	3	1	6
	LP	7	36	0	0	0	0	0
	RP	14	4	89	0	0	1	0
	LH-ca	6	0	1	21	0	5	1
	LH-cu	0	1	1	0	14	0	2
	RH-ca	4	0	0	4	0	45	1
	RH-cu	0	0	0	0	1	1	10

*L, left; R, right; P, posterior semi-circular canal; H, horizontal semi-circular canal; ca, canalolithiasis; cu, cupulolithiasis.*

**TABLE 4:** Summary results of the model in diagnosing types of benign paroxysmal positional vertigo (BPPV).

Number	TPR/ Recall	FPR	ACC	TNR	Precision	F1-scores
502	0.8848	0.1159	0.8845	0.8841	0.8981	0.8914

*ACC, accuracy; TPR (sensitivity), true positive rate; FPR, false-positive rate; TNR (specificity), true negative rate.*

## Discussion

In this study, we created a multidimensional BPPV diagnosis system with a sensitivity of 0.8848 and specificity of 0.8841, based on deep learning models. Poor specialist referral rates and the limited sensitivity of nystagmus detection with the naked eye have led to the delayed diagnosis and mismanagement of vertigo, which may both significantly impact individual health and a heavy burden on primary care (Lopez-Escamez et al., 2005; Wang et al., 2014).

### Previous Work

Previous studies have investigated the automatic detection of nystagmus, while an entire AI-based BPPV diagnosis system has not been implemented. Zhang et al. (2021) proposed a model for torsional BPPV nystagmus based on optical flow techniques which could effectively avoid the disturbance due to eyelash occlusion and pupil deformation. However, this model only supplied a basal framework for torsional nystagmus detection and could not be directly applied in disease diagnosis. Lim et al. (2019) developed a diagnostic decision support system for BPPV diagnosis using a 2D-CNN model. They showed that this system could predict the affected canals with high sensitivity and specificity with a large amount of training data, while this was limited when annotated data by otologic experts was insufficient. Newman et al. (2021) proposed an 1D-CNN model to predict nystagmus from corner-retinal potentials captured by the continuous ambulatory vestibular assessment (CAVA) device. This method was annotative and effective; however, it is not feasible for torsional nystagmus and also not acceptable for short-time positional tests (since patients have to wear CAVA device for a long time).

### Improvements

Our study was specifically designed to address the limitations of these previous studies. Thus, we generated a complete system that refined eye movement velocity curves from raw clinic test videos, trained deep learning models to predict horizontal/vertical/torsional nystagmus, and automatically diagnosed BPPV diseases using quantitative metrics. Moreover, our system is interpretable, and the accessibility of data (e.g., eye movement time-series, torsional movement images, quantitative metrics) generated in each procedure of our system is important in the medical field.

The article "A Deep Learning Model for Three-Dimensional Nystagmus Detection and Its Preliminary Application" was retracted in 2023. Reasons: compromised peer review; unreliable results or conclusions.

The BPPV detection system developed in our study can automatically detect horizontal/torsional/vertical nystagmus and BPPV diseases with a high AUC, F1-score, sensitivity, and specificity. The AUC is an overall measure of accuracy that combines sensitivity and specificity into a single metric. Our nystagmus detection model obtained good AUCs in both horizontal and torsional directions (Table 2). However, in terms of automatic BPPV diagnosis, the AUC was not reliable because of the class imbalances in our patient distribution. Data are said to be class imbalanced when the class distributions are highly imbalanced. For these multi-class cases, without loss of generality, the minority class is usually very infrequent. If one applies traditional classifiers on the dataset, the model would prefer to predict everything as negative (majority class), which was regarded as a serious problem in learning from highly imbalanced datasets. Therefore, F1 scores, sensitivity, and specificity are more suitable for sparse multi-label situations. We found a sensitivity of 0.8848, specificity of 0.8841, and F1 score of 0.8914 in final BPPV diagnosis (Tables 3, 4).

The improvement of our torsional movement detection method, compared with previous work, (Ong and Haslwanter, 2010; Jin et al., 2020; Zhang et al., 2021) can be attributed to the implementation of several image processing techniques. We first adopted the log-polar transformation to extract iris features, then applied phase correlation techniques to measure the shift between each frame. Subsequently, the torsional nystagmus signals could be obtained from the movement pattern of the iris, which is acceptable for deep learning model training.

Techniques mentioned in previous studies (Ong and Haslwanter, 2010; Jin et al., 2020; Zhang et al., 2021) belong to two main categories. The first type of technique involves extraction of iris feature points and then using them to calculate the displacement of the iris based on the correspondence of the feature points between the two frames of images, such as the optical flow method. The second type of technique involves the use of a feature similarity comparison, such as the Oriented FAST and Rotated BRIEF algorithm, image pixel histogram comparison, and template matching, to find the displacement angle of the iris when the maximum similarity occurs based on the comparison information obtained between the target and the reference image. However, feature extraction is essentially the extraction of texture information of the iris, which is highly susceptible to the influence of eyelids, reflections, and other factors. Therefore, manual processing of noise points is required, and this manual scheme cannot be applied to frame-by-frame recognition of videos. Our method makes two improvements to the previous algorithms based on template matching. First, the logarithmic polar coordinate transform is used instead of the original linear polar coordinate transform, which can better restore the iris texture features. Second, the phase correlation method is used instead of the original stencil-matching method. The phase correlation method can provide an offset in two dimensions and focus more on extracting the overall iris information. It is more robust than pixel-level schemes such as template matching and optical flow.

The article "A Deep Learning Model for Three-Dimensional Nystagmus Detection and Its Preliminary Application" was retracted in 2023. Reasons: compromised peer review; unreliable results or conclusions.

Another technical improvement in our study was the implementation of a deep learning model in pupil detection, based on previous work. General approaches for pupil detection rely on computer vision methods such as edge detection, intensity thresholding, and intensity gradient distribution, which are not feasible here due to the irregular eye movement, fast head-turning, and image processing challenges (e.g., reflections, eyelid closure, video blurring). Some previous work (Santini et al., 2018; Eivazi et al., 2019) shows the outstanding performance on pupil detection using deep learning models. In this study, we applied an object detection model to localise a patient’s pupil in a clinical video. We pre-trained a pupil detection model on a public pupil dataset (Tonsen et al., 2016) and then transferred the model to our private datasets.

The diagnosis of BPPV is based on the different characteristics of the nystagmus elicited by the provoking manoeuvres (Pérez-Vázquez and Franco-Gutiérrez, 2017). The comprehensive diagnosis of BPPV includes the specification of the affected semi-circular canal(s) and pathophysiology (canalolithiasis or cupulolithiasis) (Von Brevern et al., 2015). Our model can identify different types of nystagmus and provide the complete diagnosis of BPPV, although some rare variants of BPPV, such as canalolithiasis of the anterior canal (AC-BPPV) and cupulolithiasis of the posterior canal (PC-BPPV-cu), were not presented in our results due to the limited number of patients with these diseases. Since the model achieved high accuracy and sensitivity in BPPV diagnosis, the automated diagnostic support system based on our model could greatly benefit BPPV patients in primary care practice or emergency departments. Moreover, our model can be widely applied in various scenarios when embedded in mobile phones or other devices for eye tracking. As for the target population and clinical application, we attempted to identify nystagmus in all patients with vertigo, not only those with BPPV disease (Lim et al., 2019; Newman et al., 2021; Zhang et al., 2021).

The article "A Deep Learning Model for Three-Dimensional Nystagmus Detection and Its Preliminary Application" was retracted in 2023. Reasons: compromised peer review; unreliable results or conclusions.

Nystagmus and other nystagmus-like movements are important signals for identifying whether a patient has vestibular and neurological disorders (Eggers et al., 2019). Detailed examinations of eye movements have been shown to play a key role in differentiating between central and peripheral vertigo (Kattah et al., 2009; Brandt and Dieterich, 2017; Pudszuhn et al., 2020). Our system can identify irregular non-BPPV nystagmus, including upbeat and downbeat nystagmus, indicating different pathologies and helping in clinical diagnosis and treatment. Additionally, we can extract and quantify all parameters of nystagmus, which allows for the objective assessment of prognosis and therapeutic efficacy in patients with vertigo. Considering its complexity and pronounced individual heterogeneity, our system could provide new insights into subtype identification. It is worth noting that this system can only provide a reference diagnosis for limited categories of vertigo, raising the need for further understanding of vertigo pathophysiology and a comprehensive system with various clinical characteristics. Thus, our system provides a solid basis for further research.

### Limitations

Our study has several limitations. First, this system was developed and optimised with data obtained from a single centre; thus, it requires further validation and optimisation based on large-scale data from multiple centres in the future. Second, there are currently no standardised algorithms or open-source datasets for BPPV diagnosis, meaning that it is difficult to set a benchmark for model evaluation. Moreover, due to the privacy restrictions of clinical data, it is problematic for our model to be widely tested on other datasets. The third limitation was the DC drift of the signal. Positional tests usually last for several minutes, with the continuous movement of the patient’s pupil. We applied several methods to counteract this, including using the velocity signal instead of displacement, reducing the input length of the time-series, and consistently tracing the pupil centre as the coordinate origin. However, the accuracy of the model is still affected, especially in torsional nystagmus detection.

The article "A Deep Learning Model for Three-Dimensional Nystagmus Detection and Its Preliminary Application" was retracted in 2023. Reasons: compromised peer review; unreliable results or conclusions.

### Conclusion

In summary, we developed an automated, interpretable, and validated system that performs real-time video quality feedback, pupil location, iris torsion measurement, data augmentation, nystagmus detection, and disease inference. With these functions, the system can provide a clinical reference and facilitate nystagmus detection and diagnosis. Hence, the proposed method can be applied in real-world medical practice.

## Data Availability Statement

The raw data supporting the conclusions of this article will be made available by the authors, without undue reservation.

## Ethics Statement

The studies involving human participants were reviewed and approved by the Ethics Committee of Shanghai Sixth People’s Hospital. The patients/participants provided their written informed consent to participate in this study.

## Author Contributions

DY, YZ, and HS contributed to the conceptualisation, funding acquisition, and writing—review and editing. ZC, YF, HW, QL, and JL contributed to the investigation and resources. YW, JP, and LG contributed to the software. WL, ZL, and YL contributed to the writing – original draft, methodology, project administration, and validation. SY supervised the study. All authors contributed to the article and approved the submitted version.

## Conflict of Interest

YW, JP, and LG were employed by IceKredit Inc. The remaining authors declare that the research was conducted in the absence of any commercial or financial relationships that could be construed as a potential conflict of interest.

## Publisher’s Note

All claims expressed in this article are solely those of the authors and do not necessarily represent those of their affiliated organizations, or those of the publisher, the editors and the reviewers. Any product that may be evaluated in this article, or claim that may be made by its manufacturer, is not guaranteed or endorsed by the publisher.

## References

[B1] Abdullah-Al-WadudM.KabirM. H.Akber DewanM. A.ChaeO. (2007). “A dynamic histogram equalization for image contrast enhancement,” in *Proceedings of the 25th IEEE International Conference on Consumer Electronics*, (Piscataway, NJ: IEEE), 435. 10.1109/ICCE.2007.341567

[B2] AlbaA.Aguilar-PonceR. M.Vigueras-GomezJ. F.Arce-SantanaE. (2013). “Phase correlation based image alignment with subpixel accuracy. advances in artificial intelligence,” in *Proceedings of the 11th Mexican International Conference on Artificial Intelligence, MICAI 2012*, eds BatyrshinI.González MendozaM. (Berlin: Springer), 171–182. 10.1007/978-3-642-37807-2_15

[B3] AlyonoJ. C. (2018). Vertigo and dizziness: understanding and managing fall risk. *Otolaryngol. Clin. North Am.* 51 725–740. 10.1016/j.otc.2018.03.003 29803531

The article "A Deep Learning Model for Three-Dimensional Nystagmus Detection and Its Preliminary Application" was retracted in 2023. Reasons: compromised peer review; unreliable results or conclusions.

[B4] AraujoH.DiasJ. M. (1997). “An introduction to the log-polar mapping image sampling,” in *Proceedings II Workshop on Cybernetic Vision (Cat. No.96TB)*, (Sao Carlos), 139–144.

[B5] BhansaliS. A.HonrubiaV. (1999). Current status of electronystagmography testing. *Otolaryngol. Head. Neck Surg.* 120 419–426. 10.1016/S0194-5998(99)70286-X 10064649

[B6] BrandtT.DieterichM. (2017). The dizzy patient: don’t forget disorders of the central vestibular system. *Nat. Rev. Neurol.* 13 352–362. 10.1038/nrneurol.2017.58 28429801

[B7] EggersS. D. Z.BisdorffA.Von BrevernM.ZeeD. S.KimJ. S.Perez-FernandezN. (2019). Classification of vestibular signs and examination techniques: nystagmus and nystagmus-like movements. *J. Vestib. Res.* 29 57–87. 10.3233/VES-190658 31256095PMC9249296

[B8] EggertT. (2007). Eye movement recordings: methods. *Dev. Ophthalmol.* 40 15–34. 10.1159/000100347 17314477

[B9] EivaziS.SantiniT.KeshavarziA.KublerT.MazzeiA. (2019). “Improving real-time CNN-based pupil detection through domain-specific data augmentation,” in *Proceedings of the 11th ACM Symposium On Eye Tracking Research and Applications (ETRA)* (New York, NY). 10.1145/3314111.3319914

[B10] GanançaM. M.CaovillaH. H.GanançaF. F. (2010). Electronystagmography versus videonystagmography. *Braz. J. Otorhinolaryngol.* 76 399–403. 10.1590/S1808-8694201000030002120658023PMC9442181

[B11] HanleyK.O’dowdT.ConsidineN. (2001). A systematic review of vertigo in primary care. *Br. J. Gen. Pract.* 51 666–671. 11510399PMC1314080

[B12] JinN.MavromatisS.SequeiraJ.CurcioS. (2020). A robust method of eye torsion measurement for medical applications. *Information* 11:408. 10.3390/info11090408

[B13] KatsarkasA. (1999). Benign paroxysmal positional vertigo (BPPV): idiopathic versus post-traumatic. *Acta Otolaryngol.* 119 745–749. 10.1080/00016489950180360 10687929

[B14] KattahJ. C.TalkadA. V.WangD. Z.HsiehY. H.Newman-TokerD. E. (2009). HINTS to diagnose stroke in the acute vestibular syndrome: three-step bedside oculomotor examination more sensitive than early MRI diffusion-weighted imaging. *Stroke* 40 3504–3510. 10.1161/STROKEAHA.109.551234 19762709PMC4593511

[B15] KovacsE.WangX.GrillE. (2019). Economic burden of vertigo: a systematic review. *Health Econ. Rev.* 9:37. 10.1186/s13561-019-0258-2 31883042PMC6933936

[B16] KruschinskiC.KerstingM.BreullA.KochenM. M.KoschackJ.Hummers-PradierE. (2008). [Frequency of dizziness-related diagnoses and prescriptions in a general practice database]. *Z Evid. Fortbild Qual. Gesundhwes.* 102 313–319. 10.1016/j.zefq.2008.05.001 19006919

[B17] LimE. C.ParkJ. H.JeonH. J.KimH. J.LeeH. J.SongC. G. (2019). Developing a diagnostic decision support system for benign paroxysmal positional vertigo using a deep-learning model. *J. Clin. Med.* 8:633. 10.3390/jcm8050633 31072056PMC6571642

The article "A Deep Learning Model for Three-Dimensional Nystagmus Detection and Its Preliminary Application" was retracted in 2023. Reasons: compromised peer review; unreliable results or conclusions.

[B18] Lopez-EscamezJ. A.GamizM. J.Fernandez-PerezA.Gomez-FiñanaM. (2005). Long-term outcome and health-related quality of life in benign paroxysmal positional vertigo. *Eur. Arch. Otorhinolaryngol.* 262 507–511. 10.1007/s00405-004-0841-x 15942805

[B19] MaarsinghO. R.DrosJ.SchellevisF. G.Van WeertH. C.BindelsP. J.HorstH. E. (2010a). Dizziness reported by elderly patients in family practice: prevalence, incidence, and clinical characteristics. *BMC Fam. Pract.* 11:2. 10.1186/1471-2296-11-2 20064231PMC2817676

[B20] MaarsinghO. R.DrosJ.SchellevisF. G.Van WeertH. C.Van Der WindtD. A.Ter RietG. (2010b). Causes of persistent dizziness in elderly patients in primary care. *Ann. Fam. Med.* 8 196–205. 10.1370/afm.1116 20458102PMC2866716

[B21] MurdinL.SchilderA. G. (2015). Epidemiology of balance symptoms and disorders in the community: a systematic review. *Otol. Neurotol.* 36 387–392. 10.1097/MAO.0000000000000691 25548891

[B22] NeuhauserH. K. (2016). The epidemiology of dizziness and vertigo. *Handb. Clin. Neurol.* 137 67–82. 10.1016/B978-0-444-63437-5.00005-4 27638063

[B23] NeuhauserH. K.Von BrevernM.RadtkeA.LeziusF.FeldmannM.ZieseT. (2005). Epidemiology of vestibular vertigo: a neurotologic survey of the general population. *Neurology* 65 898–904. 10.1212/01.wnl.0000175987.59991.3d 16186531

[B24] NewmanJ. L.PhillipsJ. S.CoxS. J. (2021). 1D convolutional neural networks for detecting nystagmus. *IEEE J. Biomed. Health Inform.* 25 1814–1823. 10.1109/JBHI.2020.3025381 32956068

[B25] OjansivuV.HeikkilaJ. (2007). Image registration using blur-invariant phase correlation. *IEEE Signal Proc. Lett.* 14 449–452. 10.1109/LSP.2006.891338 23782811

[B26] OngJ. K. Y.HaslwanterT. (2010). Measuring torsional eye movements by tracking stable iris features. *J. Neurosci. Methods* 192 261–267. 10.1016/j.jneumeth.2010.08.004 20708033PMC2958308

[B27] Pérez-VázquezP.Franco-GutiérrezV. (2017). Treatment of benign paroxysmal positional vertigo, a clinical review. *J. Otol.* 12 165–173. 10.1016/j.joto.2017.08.004 29937852PMC6002633

[B28] PudszuhnA.HeinzelmannA.SchönfeldU.NiehuesS. M.HofmannV. M. (2020). [Acute vestibular syndrome in emergency departments : clinical differentiation of peripheral and central vestibulopathy]. *Hno* 68 367–378. 10.1007/s00106-019-0721-8 31440773

[B29] ReddyB. S.ChatterjiB. N. (1996). An FFT-based technique for translation, rotation, and scale-invariant image registration. *IEEE Trans. Image Proc.* 5 1266–1271. 10.1109/83.506761 18285214

[B30] SantiniT.FuhlW.KasneciE. (2018). “PuReST: robust pupil tracking for real-time pervasive eye tracking,” in *Proceedings of the ACM Symposium on Eye Tracking Research and Applications (ETRA)* (New York, NY). 10.1145/3204493.3204578

The article "A Deep Learning Model for Three-Dimensional Nystagmus Detection and Its Preliminary Application" was retracted in 2023. Reasons: compromised peer review; unreliable results or conclusions.

[B31] SchappertS. M. (1992). National ambulatory medical care survey: 1989 summary. *Vital Health Stat* 13 1–80.1376543

[B32] SzegedyC.IoffeS.VanhouckeV.AlemiA. A. (2017). “Inception-v4, inception-ResNet and the impact of residual connections on learning,” in *Proceedings of the 31st AAAI Conference on Artificial Intelligence*, (San Francisco, CA), 4278–4284.

[B33] SzegedyC.LiuW.JiaY. Q.SermanetP.ReedS.AnguelovD. (2015). “Going deeper with convolutions,” in *Proceedings of the IEEE Conference on Computer Vision and Pattern Recognition (CVPR)*, (Boston, MA), 1–9. 10.1109/CVPR.2015.7298594

[B34] TonsenM.ZhangX. C.SuganoY.BullingA. (2016). “Labelled pupils in the wild: a dataset for studying pupil detection in unconstrained environments,” in *Proceedings of the 9th Biennial ACM Symposium on Eye Tracking Research and Applications (ETRA)* (New York, NY), 139–142. 10.1145/2857491.2857520

[B35] TyrrellJ.WhinneyD. J.TaylorT. (2016). The cost of Ménière’s disease: a novel multisource approach. *Ear. Hear.* 37 e202–e209. 10.1097/AUD.0000000000000264 26760200

[B36] Von BrevernM.BertholonP.BrandtT.FifeT.ImaiT.NutiD. (2015). Benign paroxysmal positional vertigo: diagnostic criteria. *J. Vestib. Res.* 25 105–117. 10.3233/VES-150553 26756126

[B37] WainbergM.MericoD.DelongA.FreyB. J. (2018). Deep learning in biomedicine. *Nat. Biotechnol.* 36 829–838. 10.1038/nbt.4233 30188539

[B38] WangH.YuD.SongN.SuK.YinS. (2014). Delayed diagnosis and treatment of benign paroxysmal positional vertigo associated with current practice. *Eur. Arch. Otorhinolaryngol.* 271 261–264. 10.1007/s00405-012-2333-8 23455578

[B39] WolbergG.ZokaiS. (2000). “Robust image registration using log-polar transform,” in *Proceedings of the IEEE International Conference on Image Processing (ICIP 2000)*, (Vancouver, BC), 493–496. 10.1109/ICIP.2000.901003

[B40] YaoQ.WangH.SongQ.ShiH.YuD. (2018). Use of the Bárány Society criteria to diagnose benign paroxysmal positional vertigo. *J. Vestib. Res.* 28 379–384. 10.3233/VES-190648 30814370

[B41] YildirimO.PlawiakP.TanR. S.AcharyaU. R. (2018). Arrhythmia detection using deep convolutional neural network with long duration ECG signals. *Comput. Biol. Med.* 102 411–420. 10.1016/j.compbiomed.2018.09.009 30245122

[B42] ZabihiM.RadA. B.KiranyazS.SarkkaS.GabboujM. (2019). 1D convolutional neural network models for sleep arousal detection. *arXiv* [Preprint] arXiv:1903.01552, 31946784

[B43] ZhangW. L.WuH. Y.LiuY.ZhengS.LiuZ. Z.LiY. R. (2021). Deep learning based torsional nystagmus detection for dizziness and vertigo diagnosis. *Biomed. Signal Proc. Control* 68:102616. 10.1016/j.bspc.2021.102616

